# *FCGR2A* Could Function as a Prognostic Marker and Correlate with Immune Infiltration in Head and Neck Squamous Cell Carcinoma

**DOI:** 10.1155/2021/8874578

**Published:** 2021-07-05

**Authors:** Yongmei Dai, Wenhan Chen, Junpeng Huang, Tongjian Cui

**Affiliations:** ^1^Department of Oncology, Shengli Clinical Medical College of Fujian Medical University & Fujian Provincial Hospital, Fujian 350001, China; ^2^The Second Clinical Medical College of Fujian Medical University, Fujian 362000, China

## Abstract

**Objective:**

We aim to investigate the correlation between *FCGR2A* mRNA level and prognosis of head and neck squamous cancer (HNSC) in public databases. In addition, we investigated the correlation between *FCGR2A* expression and clinicopathological characteristics and tumor-infiltrating immune cells in HNSC patients.

**Methods:**

*FCGR2A* mRNA expression in multiple cancers was analyzed based on Gene Expression Profiling Interactive Analysis. A protein-protein interaction network was obtained based on the STRING database. The 10 proteins most closely related to FCGR2A (i.e., CD3G, PLCG2, LAT, LYN, SYK, FCGR3A, PIK3R1, HCK, ITGAM, and ITGB2) were screened, followed by establishing the protein-protein interaction network. The correlation between *FCGR2A* expression and immunocytes was investigated, together with the effects of FCGR2A on the metastasis, recurrence, and survival of HNSC.

**Results:**

*FCGR2A* expression in several carcinoma tissues was significantly higher than that of adjacent tissues. Significant differences were noticed in the HNSC samples and the adjacent tissue samples except the seven samples of grade 4. There were statistical differences between the *FCGR2A* expression in tissues of grade 1, grade 2, and grade 3 (*P* < 0.05). In the tissues of grade 4, the expression of FCGR2A was the lowest. The FCGR2A protein was a type of II-a receptor in *γ*Fc of the low-affinity immunoglobulin, which could bind with the Fc region of the immunoglobulin *γ*. There was a correlation between the *FCGR2A* gene and the distal HNSC metastasis. *FCGR2A* gene expression was correlated with the survival and prognosis. The GSE65858 dataset was selected for the validation. The *FCGR2A* expression was significantly correlated with total survival (*P* = 0.0107) and progression-free survival (*P* = 0.0362).

**Conclusions:**

Our findings shed light on the importance of *FCGR2A* in HNSC and illustrated a potential relationship between *FCGR2A* and tumor-immune interactions.

## 1. Introduction

Head and neck squamous cancer (HNSC), one of the most common types of human malignancy, shows an annual incidence of more than 780,000 cases worldwide [1–3]. To date, the treatment options of HNSC include surgery, radiation, and chemotherapy; however, it leads to a mortality rate of up to 50% [4]. Currently, most of the studies on HNSC are mainly focused on disease prevention, early screening, identification of target molecules, and the establishment of new therapies. To our best knowledge, there are still some disadvantages in the prediction of prognosis among HNSC patients. Therefore, it is urgent to screen specific and sensitive biomarkers for the evaluation of an individualized treatment regimen.

The *FCGR2A* gene, responsible for encoding the Fc*γ*RIIa protein, is localized at 1q23 [5] consisting of 10 exons and 9 introns. It is a member of the immunoglobulin Fc receptor (FCGR) gene on the surface of cells involved in immune responses. Based on its function, Fc*γ*RIIa is divided into two subtypes including Fc*γ*RIIa and Fc*γ*RIIb, which are classified as IgG receptors with low to moderate affinity. It is mainly involved in binding with IgG, and is expressed in the neutrophils, monocytes, macrophages, dendritic cells (DCs), B lymphocytes, and platelets. In a previous study, FCGRs generated by the natural killer (NK) cells, macrophages, and DCs could modulate the antibody-dependent cytotoxicities, which were crucial for the elimination of cancer cells. *FCGR2A* gene polymorphism was reportedly associated with the susceptibility of inflammation-related diseases, such as atherosclerosis [6], Takayasu arteritis [7], systemic lupus erythematosus (SLE) [8], and ulcerative colitis [9]. To date, some studies have been conducted to investigate the roles of *FCGR2A* gene polymorphism in malignancies. In a previous study [10], the *FCGR2A* genotype was associated with the treatment efficiency of colorectal cancer patients who received cetuximab administration, which triggered no additional toxicities. To our best knowledge, few studies focused on the investigation on the oncogenic roles of the *FCGR2A* gene in HNSC in a systematic manner. In this study, we evaluated the association between *FCGR2A* mRNA level and HNSC prognosis in public databases such as TCGA, TISCH, Exocarta, and CPTAC. Moreover, we investigated the correlation between *FCGR2A* expression and clinicopathological characteristics or the tumor-infiltration in HNSC patients. Our findings shed light on the importance of *FCGR2A* in HNSC and contributed to the investigation on the potential relationship between *FCGR2A* and tumor-immune interaction and its underlying mechanism.

## 2. Materials and Methods

### 2.1. Expression of *FCGR2A* mRNA

The Human Protein Atlas database (http://www.proteinatlas.org/) was utilized to analyze the expression of *FCGR2A* in multiple cancers. In addition, the expression profile of the mRNA and protein in the normal tissues and cells was analyzed. Gene Expression Profiling Interactive Analysis (GEPIA, http://gepia.cancer-pku.cn/) was utilized to analyze the expression differences of *FCGR2A* in different cancers and the adjacent cancer tissues, followed by depicting the plot. Moreover, the expression of *FCGR2A* in HNSC was explored using UALCAN dataset (http://ualcan.path.uab.edu) based on the gender, age, and other classification standards.

### 2.2. FCGR2A Protein Interaction Network and the Gene Enrichment Analysis

The protein-protein interaction network was obtained based on the STRING database. On this basis, the top 10 proteins related to FCGR2A (CD3G, PLCG2, LAT, LYN, SYK, FCGR3A, PIK3R1, HCK, ITGAM, and ITGB2) were screened, followed by establishing the protein-protein interaction network. In the homepage of Metascape (http://metascape.org), enrichment analysis was performed after entering the 11 genes including *FCGR2A*, *CD3G*, *PLCG2*, *LAT*, *LYN*, *SYK*, *FCGR3A*, *PIK3R1*, *HCK*, *ITGAM*, and *ITGB2*. Then, KEGG pathway analysis, GO analysis, and gene sets were integrated and visualized. Finally, the 11 genes encoding these proteins including FCGR2A were entered into Metascape.

### 2.3. Correlation between *FCGR2A* Expression and Immunocytes

The TIMER database [11] (http://cistrome.dfci.harvard.edu/TIMER/) was utilized to determine the association between *FCGR2A* expression and the immune infiltration. To begin with, the purity estimation was acquired using the tool CHAT [12] and validated by a diluted series with known tumor/normal mixture ratios. On this basis, we established the correlation between *FCGR2A* expression and tumor purity. Pearson's correlation was utilized for the analysis. Next, *FCGR2A-*expressing tumors in HNSC showed various immunocyte infiltration levels, including B lymphocytes, CD4+ T lymphocytes, CD8+ T lymphocytes, neutrophils, macrophages, and DCs.

### 2.4. Effects of *FCGR2A* on the Metastasis, Recurrence, and Survival of HNSC

To investigate the prognostic role of *FCGR2A* mRNA in HNSC, the Kaplan-Meier plotter [13] (http://www.kmplot.com) was used to determine the prognostic significance. Based on the GEOquery package, the HNSC GSE65858 was downloaded from the GEO database [14] for the prognosis analysis. There were 253 tumor samples in the GSE65858 database, among which 179 were human papilloma virus- (HPV-) negative samples. The sequencing platform was Illumina HumanHT-12 v4.0. Downloaded from The Cancer Genome Atlas (TCGA) database, the Long-term Outcome and Gene Expression Profiling Database of Pancancer (LOGpc) platform was used for analyzing the overall survival (OS) and disease-free survival (DSS) of HNSC patients.

### 2.5. Statistical Analysis

Kaplan-Meier method was used for estimating the survival curve. To compare the survival curve, the log-rank test was utilized for the hazard ratio (HR) and the *P* value of the Kaplan-Meier plotter and GEPIA. Spearman's analysis was utilized for the analysis of the correlation of genes.

## 3. Results

### 3.1. Expression of *FCGR2A* mRNA

According to the Human Protein Atlas website, the *FCGR2A* gene was expressed in various tissues. Serum *FCGR2A* mRNA was the highest among these tissues (Figure 1). The enriched cell types of the blood expressing the *FCGR2A* gene included neutrophils, eosinophils, and monocytes (Figure 2). In the cellular views, *FCGR2A* was mainly expressed in the Golgi body and the cell membrane (Figure 3).

In the GEPIA website, we compared the expression of *FCGR2A* in the adjacent cancer tissues and the cancer tissues. Expression of *FCGR2A* in the carcinoma of the bile duct, carcinoma of the esophagus, the glioblastoma multiforme, HNSC, the clear cell carcinoma of the kidney, renal papillary cell carcinoma, low-grade cerebral glioma, ovary serous cystadenocarcinoma, carcinoma of the pancreas, melanoma, and gastric cancer tissues was significantly higher than that of the corresponding adjacent tissues. In contrast, the expression of *FCGR2A* in the adrenocortical carcinoma, diffuse large B cell lymphoma, acute myeloid leukemia, pulmonary squamous carcinoma, and thymus cancer tissues was significantly lower than that of the corresponding adjacent tissues (Figure 4).

### 3.2. Expression of *FCGR2A* in HNSC

We compared the HNSC samples with the adjacent tissues based on the UALCAN website and tried to investigate the correlation between *FCGR2A* expression and the clinicopathological factors. As shown in Figure 5, significant differences were noticed in the HNSC samples and the adjacent tissue samples except the seven samples of grade 4, based on various clinicopathological factors. Compared with HPV-positive samples, the *FCGR2A* expression in the HPV-negative HNSC patients showed a significant increase (*P* < 0.05). The expression of *FCGR2A* was associated with the tumor grading, in a grade-dependent manner. There were statistical differences between the *FCGR2A* expression in tissues of grade 1, grade 2, and grade 3 (*P* < 0.05). In the tissues of grade 4, the expression of *FCGR2A* was the lowest. However, there were only seven samples, and we could not evaluate the reliability of the results. There were no statistical differences in the expression of *FCGR2A* among the samples obtained from cases of different gender, race, and tumor staging (*P* > 0.05).

### 3.3. FCGR2A Protein Interaction Network and Gene Enrichment Analysis

Upon entry of FCGR2A into the STRING website, the gene database of *Homo sapiens* was selected. The data indicated that the FCGR2A protein was a type of II-a receptor in the *γ*Fc of the low-affinity immunoglobulin, which could bind with the Fc region of the immunoglobulin *γ*. It could promote the phagocytosis of the antigens. Besides, it triggered the cellular responses targeting the pathogens and soluble antigens through binding with the IgG.

We then screened the top 10 proteins that were closely related to FCGR2A including CD3G, PLCG2, LAT, LYN, SYK, FCGR3A, PIK3R1, HCK, ITGAM, and ITGB2. On this basis, the protein-protein interaction network was established (Figure 6). Subsequently, the genes encoding the 11 proteins including the top 10 proteins and the FCGR2A protein were entered into the Metascape website, using *H. sapiens* as the type. Initially, we confirmed all the enriched items that were subject to statistical analysis, such as GO/KEGG, the typical signaling pathway, and hallmark gene sets. The enriched plot was obtained based on the *P* value and enriched factors (Figure 7). Afterwards, the enrichment plot was transmitted to the network topology. Each item was represented by a circle node. Its size was positively correlated to the gene amount. The items with a similarity score of >0.3 were linked by a line, of which the line thickness represented the similarity score (Figure 8).

### 3.4. Correlation between Expression of *FCGR2A* and Immunocytes in TIMER

In this study, the TIMER database was utilized to investigate the correlation between *FCGR2A* expression and immune infiltration of HNSC (Table 1). The scatter plot displayed the corrected partial Spearman's correlation and the statistical significance. On this basis, there was a negative correlation between *FCGR2A* expression and the HNSC purity. Meanwhile, there were significant differences in the 6 types of immunocytes and *FCGR2A* expression (*P* < 0.05), especially the DCs, neutrophils, and macrophages. There was a correlation between *FCGR2A* expression and the 6 infiltrating immunocytes regardless of the HPV negativity or positivity (Figure 9). This implied that *FCGR2A* expression was correlated with the immune infiltration of HNSC.

The SCNA model was utilized to explore the association between the *FCGR2A* gene copy number variation (CNV) and the richness of the immune infiltration. Based on the CNA, we determined the infiltration of 6 types of immunocytes. GISTIC 2.0 served as the grouping standards for the CNA which were divided into 5 types including deep deletion (-2), arm-level deletion (-1), diploid/normal (0), arm-level gain (1), and high amplification (2). Except the CD4+ T lymphocytes from the HPV-negative samples, there was a significant correlation between the *FCGR2A* expression and arm deletion in the immunocytes in all the HNSC samples and HPV-negative HNSC samples. In contrast, there was no correlation between the *FCGR2A* expression and arm deletion in the immunocytes between all the HNSC samples and HPV-positive HNSC samples. As shown in Figure 10, the infiltration of DCs was higher in the cells with no anomaly in the chromosome structure or those with enlarged arms.

To further investigate the correlation between *FCGR2A* and various immune infiltration cells, TIMER was used to investigate the correlation between *FCGR2A* expression and the immune-labeled genes (Table 2) in B lymphocytes, T lymphocytes, NK cells, DCs, macrophages, monocytes, neutrophils, eosinophils, basophils, mastocytes, platelets, megakaryocytes, and red blood cells. Our data showed that *FCGR2A* expression was correlated with the expression of 21 immune markers in the HNSC samples. In the adjacent cancer tissues, the expression of *FCGR2A* was correlated with 16 immune markers.

### 3.5. Roles of *FCGR2A* Gene in the Evaluation of HNSC Prognosis

In this section, PROGgene V2 was used for the correlation between the *FCGR2A* gene and the distal metastasis or local recurrence in the HNSC samples. These data indicated a correlation between the *FCGR2A* gene and distal HNSC metastasis (*P* = 0.012). In contrast, there was no correlation between local recurrence and the expression of the *FCGR2A* gene (*P* = 0.13, Figure 11).

Subsequently, the LOGpc database was used for analyzing the survival of HNSC patients, followed by analysis of TCGA data. This indicated that the *FCGR2A* gene expression was correlated with survival and prognosis (Figure 12). To be specific, there were statistical differences in the survival probability between the high *FCGR2A* mRNA samples and low *FCGR2A* mRNA samples. Meanwhile, the GSE65858 dataset was selected for the validation. The FCGR2A expression was significantly correlated with total survival (*P* = 0.0107) and progression-free survival (*P* = 0.0362, Figure 13). This further validated that expression of *FCGR2A* was correlated with survival and prognosis of HNSC patients.

## 4. Discussion

A majority of HNSC patients are diagnosed at the locally advanced stages of III and IV [15]. In clinical settings, the main treatment option of HNSC is the combination of surgical resection and adjuvant radiotherapy, or concurrent radiotherapy and chemotherapy [16, 17]. Tumor staging and pathology analysis are crucial for the prognostic prediction, which is also an important basis for the guidance of the optimal adjuvant therapy. To date, there are no specific biomarkers for therapeutic strategies of HNSC. Fortunately, several biomarkers have been developed as potential factors to predict and evaluate the prognosis of patients. For instance, the Wnt/*β*-catenin pathway could inhibit cell apoptosis and promote the growth of squamous cell carcinoma. Additionally, the Wnt/*β*-catenin pathway was regulated by a variety of antagonistic genes that were differentially expressed in HNSC. This demonstrated a relationship with therapeutic sensitivity, which may serve as a potential biomarker for treatment and prognosis of HNSC [16, 18]. To date, there are still some disputes on the prognostic prediction of these biomarkers [19]. Thus, identification of independent markers associated with the prognosis of HNSC is conducive to their clinical application.

The *FCGR2A* gene encodes a member of a family of immunoglobulin Fc receptor genes that was identified on the surface of many immune response cells [20]. The FCGR2A protein is considered as a cell surface receptor on phagocytic cells (e.g., macrophages and neutrophils), which is involved in the process of phagocytosis [21]. According to the previous description, FCGR2A was mainly reported to bind with the IgG and was expressed in the neutrophils, monocytes, macrophages, and DCs [22]. Fc-gamma receptor polymorphisms were associated with efficacy but not with toxicity in wild-type KRAS, cetuximab-treated colorectal cancer patients. Additionally, in a study focused on the exploration of the influence of genetic variants on susceptibility to chronic periaortitis, Alberici et al. reported that FCGR2A was a gene hallmarker for the autoimmunity among the patients with chronic periaortitis [20]. Moreover, in a study that investigated the association of CD1 and *FCGR2A* gene polymorphisms with Guillain-Barré syndrome susceptibility, Zhang et al. indicated that *FCGR2A* gene polymorphisms may contribute to GBS risk in Caucasians and revealed a certain trend toward significance in the association of the exon 2 of the *CD1E* gene with GBS in Caucasians [23]. Up to now, there are few studies focusing on the expression of *FCGR2A* among HNSC patients. Our data showed that *FCGR2A* expression was correlated with the expression of 21 immune markers in the HNSC samples, while in the adjacent cancer tissues, the expression of *FCGR2A* was correlated with 16 immune markers. This contributed to the illustration on the roles of the *FCGR2A* gene in radiotherapy resistance among carcinomas of nasopharynx patients.

The circulating *FCGR2A* gene was comparatively higher than that of the other tissues. In the cellular level, the *FCGR2A* gene was mainly expressed on the Golgi body and the cell membrane. As revealed by the GEPIA website, *FCGR2A* level in partial cancer tissues was comparatively higher than the adjacent normal tissues, including carcinoma of bile duct, esophagus carcinoma, clear cell carcinoma of kidney, and gastric cancer. In the HNSC patients with HPV negativity, the expression of *FCGR2A* in cancer tissues was higher than that of the adjacent tissues. Paradoxically, in certain types of tumor, the expression of *FCGR2A* in the cancer tissues was significantly lower than the adjacent tissues. To date, little is known about the association between the expression of *FCGR2A* and the prognosis of these patients, as most of the studies focused on the *FCGR2A* polymorphism. In our study, the expression of *FCGR2A* mRNA and protein was reported to be associated with the tumor staging from grade 1 to grade 3. Interestingly, in those with grade 4 cancer, the expression of *FCGR2A* showed a decline in all the 7 cases. This may not present a trend as the sample size is not adequate. Besides, our data indicated that there was no correlation between *FCGR2A* expression and gender, race, and tumor staging.

In this study, we screened the top 10 proteins associated with FCGR2A, which formed a potential protein interaction network involving the activation of the FCGR signaling pathway. After network analysis, these proteins were involved in FCGR activation, immunological response activation, phagocytosis, PI3KCI signaling pathway, PTP1B signaling pathway, integrin-mediated signaling pathway, CD28 family cosimulation, and bacterial response. According to the GBM/OV microarray database in the Timer website, the expression of FCGR2A was associated with the function of 6 types of immunocytes. Then, the TIMER databases were employed to investigate the correlation between the expression of FCGR2A in the immunocytes of the HNSC patients and the expression of immune marker genes, which indicated that the *FCGR2A* gene may be involved in the immune infiltration of the HNSC. In addition, infiltration of tumor immunocytes refer to a process in which immunocytes are transmitted to the cancer tissues through circulation. On this basis, it was possible to isolate the infiltrated immunocytes from the cancer tissues. According to a previous study, the infiltration of immunocytes in cancer tissues was considered to be related to the clinical outcomes in cancer patients. Therefore, infiltration of immunocytes in cancer tissues may serve as a drug target in clinical treatment.

PROGgeneV2 is a software displaying the prognostic implications of genes in various cancers. To our best knowledge, most of the studies on FCGR2A have been focused on the inflammation and cerebral vascular diseases. For instance, in a recent study, there was variation in the expression of the *FCGR2A* gene in the platelets after onset of myocardial infarction [24]. Besides, *FCGR2A* single nucleotide polymorphism conferred susceptibility to childhood-onset idiopathic nephrotic syndrome [25]. Moreover, there was genetic variation of human neutrophil Fc*γ* receptors and SIRP*α* in antibody-dependent cellular cytotoxicity toward cancer cells [26]. In this study, it was used to investigate the correlation of *FCGR2A* gene expression and the distal metastasis and local occurrence of HNSC. The results showed that the *FCGR2A* gene was correlated with distal metastasis rather than local recurrence in HNSC patients. Subsequently, the LOGpc database was utilized to investigate the correlation between *FCGR2A* gene expression and survival of HNSC patients. These data indicated that *FCGR2A* gene expression was associated with the survival and prognosis of the HNSC patients. Based on the validation using GSE65858, there was a significant difference in the FCGR2A expression and the total survival rate of HNSC cases. Meanwhile, there was a significant association between FCGR2A expression and progression-free survival. This further validated the correlation between FCGR2A expression and the survival prognosis among HNSC patients. All these implied that *FCGR2A* may serve as an effective factor for the prediction of prognosis of HNSC.

There are some limitations in our study. We only predicted the correlation between *FCGR2A* mRNA in tumor immunology and its prognostic value based on online tools. In future, experimental studies are required to further illustrate the exact role of *FCGR2A* mRNA via downregulating or upregulating its expression.

## 5. Conclusions

In summary, our study provided insights into understanding the potential role of *FCGR2A* in tumor immunology and its prognostic value. *FCGR2A* mRNA level was correlated with prognosis and immune infiltrating levels in HNSC, which indicated that it could be used as a prognostic biomarker. In the future, further studies are required to evaluate the potency of the FCGR2A inhibitor interfering with immune cells.

## Figures and Tables

**Figure 1:** Expression of FCGR2A mRNA and protein expression in normal tissues.

**Figure 2:** FCGR2A mRNA-enriched cell types in blood samples.

**Figure 3:** Expression of *FCGR2A* in Golgi body and plasma membrane.

**Figure 4:** Expression of FCGR2A in tumor (red column) and adjacent tissues (blue column). ^∗^*P* < 0.05. ACC: adrenocortical carcinoma; BLCA: bladder urothelial carcinoma; BRCA: breast invasive carcinoma; CESC: cervical squamous cell carcinoma and endocervical adenocarcinoma; CHOL: cholangiocarcinoma; COAD: colon adenocarcinoma; DLBC: lymphoid neoplasm diffuse large B cell lymphoma; ESCA: esophageal carcinoma; GBM: glioblastoma multiforme; HNSC: head and neck squamous carcinoma; KICH: kidney chromophobe; KIRC: kidney renal clear cell carcinoma; KIRP: kidney renal papillary cell carcinoma; AML: acute myeloid leukemia; LGG: brain lower-grade glioma; LIHC: liver hepatocellular carcinoma; LUAD: lung adenocarcinoma; LUSC: lung squamous cell carcinoma; OV: ovarian serous cystadenocarcinoma; PAAD: pancreatic adenocarcinoma; PCPG: pheochromocytoma and paraganglioma; PRAD: prostate adenocarcinoma; READ: rectum adenocarcinoma; SARC: sarcoma; SKCM: skin cutaneous melanoma; STAD: stomach adenocarcinoma; TGCT: testicular germ cell tumors; THCA: thyroid carcinoma; THYM: thymoma; UCEC: uterine corpus endometrial carcinoma; UCS: uterine carcinosarcomas.

**Figure 5:** FCGR2A transcription in subgroups of patients with HNSC, stratified based on gender, race, and other criteria (UALCAN). (a) Relative expression of FCGR2A in normal and HPV-positive and HPV-negative HNSC samples. (b) Relative expression of FCGR2A in normal and HNSC patients with grade 1, 2, 3, and 4 tumors. (c) Relative expression of FCGR2A in normal or HNSC patients with stage N1, N2, N3, and N4. (d) Relative expression of FCGR2A in normal patients or in HNSC patients at stages 1, 2, 3, and 4. (e) Relative expression of FCGR2A in normal, Caucasian, African-American, and Asian HNSC patients. (f) Relative expression of FCGR2A in normal, male, and female HNSC patients. The central marker was the median; the edges of the box were the 25th and 75th percentiles. The *t*-test was used to estimate the significance of difference in gene expression levels between groups. ^∗^*P* < 0.05; ^∗∗^*P* < 0.01; ^∗∗∗^*P* < 0.001.

**Figure 6:** FCGR2A-related protein interaction network.

**Figure 7:** Heat map of enrichment of FCGR2A-related protein genes. The shade of the color depended on the *P* value.

**Figure 8:** Network diagram of enrichment of gene cluster. (a) Different colors according to enrichment item markers of different functions. (b) Different color shades according to *P* values. The size of each node was proportional to the number of input genes.

**Figure 9:** Correlation of FCGR2A expression with immune infiltration level in the TIMER database. (a) All head and neck cancer samples. (b) HPV-negative HNSC samples. (c) HPV-positive HNSC samples. The blue curve was the fitting curve of the scatter plot.

**Figure 10:** SCNA model of *FCGR2A* gene copy number variation and immunoinfiltration abundance. (a) All head and neck cancer samples. (b) HPV-negative HNSC samples. (c) HPV-positive HNSC samples. ^∗^*P* < 0.05; ^∗∗^*P* < 0.01; ^∗∗∗^*P* < 0.001.

**Figure 11:** *FCGR2A* gene expression and recurrence or metastasis curve in HNSC patients. (a) Recurrence curve. (b) Metastasis curve. Red: high gene expression; green: low gene expression.

**Figure 12:** Survival curve of *FCGR2A* gene and HNSC in TCGA samples. (a) Overall survival (OS) curve. (b) Disease-specific survival (DSS) curve.

**Figure 13:** Survival curve of *FCGR2A* gene and head and neck cancer in GSE65858 data. (a) Overall survival (OS) curve. (b) Progression-free survival (PFS) curve.

**Table 1:** Correlation between FCGR2A copy number variation and immune infiltration abundance in HNSCC.

Variable	CNA level	*P* value, HNSCC	*P* value, HNSCC-HPVneg	*P* value, HNSCC-HPVpos
B cell	Arm-level deletion	6.52*E*‐08	2.26*E*‐04	1
	Diploid/normal	1	1	1
	Arm-level gain	1.40*E*‐01	6.70*E*‐01	1.30*E*‐01
	High amplication	8.60*E*‐01	6.32*E*‐01	
CD8+ T cell	Arm-level deletion	1.33*E*‐06	9.28*E*‐05	1
	Diploid/normal	1	1	1
	Arm-level gain	4.48*E*‐05	1.64*E*‐04	6.00*E*‐02
	High amplication	3.35*E*‐01	7.26*E*‐01	
CD4+ T cell	Arm-level deletion	2.26*E*‐03	7.29*E*‐02	1
	Diploid/normal	1	1	1
	Arm-level gain	4.41*E*‐02	8.43*E*‐02	3.62*E*‐01
	High amplication	3.22*E*‐02	1.57*E*‐01	
Macrophage	Arm-level deletion	7.85*E*‐04	1.81*E*‐03	1
	Diploid/normal	1	1	1
	Arm-level gain	8.84*E*‐02	2.36*E*‐02	6.15*E*‐01
	High amplication	7.60*E*‐01	7.81*E*‐01	
Neutrophil	Arm-level deletion	6.85*E*‐03	1.20*E*‐02	1
	Diploid/normal	1	1	1
	Arm-level gain	3.85*E*‐07	1.34*E*‐05	1.57*E*‐02
	High amplication	1.50*E*‐02	1.82*E*‐02	
Dendritic cell	Arm-level deletion	5.29*E*‐05	7.38*E*‐04	1
	Diploid/normal	1	1	1
	Arm-level gain	1.17*E*‐03	1.51*E*‐02	3.78*E*‐02
	High amplication	8.90*E*‐01	9.60*E*‐01	

HNSCC: head and neck squamous cell carcinoma; HNSCC-HPVneg: HPV-negative, head and neck squamous cell carcinoma; HNSCC-HPVpos: HPV-positive, head and neck squamous cell carcinoma.

**Table 2:** Correlation between FCGR2A and immune markers of various immune cells in HNSCC tumor samples and adjacent tissues.

Immunocytes	Immune-labeled genes	HNSCC tissues		Adjacent HNSCC tissues	
		*P* value	*R*	*P* value	*R*
B lymphocytes	CD19	0.45	−0.033	0.038	0.31
T lymphocytes	CD2	5.70*E*‐13	0.31	0.22	0.19
	CD3D	6.60*E*‐06	0.2	0.14	0.22
	CD3E	6.90*E*‐11	0.28	0.22	0.19
NK cells	CD56	1.70*E*‐05	0.19	0.18	0.2
	CD94	4.20*E*‐14	0.32	0.006	0.41
	NKp46	3.60*E*‐07	0.22	0.035	0.32
Dendritic cells	CD11c	0	0.52	1.30*E*‐14	0.87
Macrophages	CD11b	1.80*E*‐07	0.23	6.20*E*‐13	0.84
	CD68	0	0.62	1.70*E*‐07	0.69
	CD163	0	0.78	1.20*E*‐10	0.79
Monocytes	CD14	0	0.73	5.10*E*‐10	0.78
Neutrophils	CD116	1.80*E*‐07	0.23	6.20*E*‐13	0.84
	CD44	8.90*E*‐10	0.26	0.12	0.24
	CD55	0.87	−0.007	0.14	0.23
Eosinophils	CD45	0	0.52	2.80*E*‐06	0.64
	CD125	0.0012	0.14	0.97	0.0061
	CD193	1.30*E*‐14	0.33	0.45	0.12
Basophils	CD22	0.99	−0.00075	0.00064	0.49
	CD45	0	0.52	2.80*E*‐06	0.64
Mastocytes	CD33	0	0.49	2.40*E*‐11	0.81
	CD117	0.00021	0.26	9.10*E*‐11	0.8
	CD203c	0.065	0.081	0.0022	0.45
Platelets	CD41	0.028	−0.096	0.78	0.043
	CD42a	0.064	0.081	0.6	0.082
	CD42b	0.7	0.017	0.0032	0.43
	CD61	0	0.45	0.00067	0.49
Megakaryocyte	CD41b	0.028	−0.096	0.78	0.043
Red blood cells	CD235a	0.27	−0.049	0.32	0.15

## Data Availability

The datasets used for the current study are available upon reasonable request from the corresponding author.
